The article "Research on the Influence of International Communication of Chinese Literature on Teenagers' Physical and Mental Health in the Digital Humanistic Environment" was retracted in 2023. Reasons: signs of a paper mill; suspected computer-generated content; unreliable results or conclusions; concerns about the data.

# Research on the Influence of International Communication of Chinese Literature on Teenagers' Physical and Mental Health in the Digital Humanistic Environment

**DOI:** 10.1155/2022/2464083

**Published:** 2022-09-28

**Authors:** Xiaoyi Wang, Ziwei Xie, Yuan Zhu

**Affiliations:** ^1^School of Languages and Communication Studies, Beijing Jiaotong University, Beijing 100044, China; ^2^School of Foreign Languages, Renmin University of China, Beijing 100872, China; ^3^School of Humanities, Tsinghua University, Beijing 100084, China

## Abstract

*Research Background*. With the enhancement of China's international influence, China has stepped into the international ecological environment in the fields of economy, politics, culture, art, and so on, accompanied by the spread of China's culture and literature. China's 5000-year-old cultural history and artistic characteristics are integrated into the ecological field of the international environment. *Research Purpose*. The international spread of Chinese literature also has a certain impact on the physical and mental health of teenagers. This paper studies and discusses the impact of international communication of Chinese literature on teenagers' physical and mental health in the digital humanistic environment. Under the development environment of Digital Humanities in China, the impact of Chinese literature on the healthy psychology of teenagers, the impact content, and the characteristics of each were evaluated. Through the comparison of physical and mental health growth of adolescents in different ages, the characteristics of physical and mental health of adolescents are explored. The coupling degree of physical and mental health of adolescents in different development environments is compared and analyzed. *Research Results*. Through the research, it is found that with the development of Digital Humanities, the spread of Chinese literature with internationalization has a positive impact on the physical and mental health and psychological quality construction of teenagers and plays a promoting role in promoting mental health, increasing personal quality, and improving teenagers' correct values. The various ideological and moral qualities of Chinese literature can play a greater role in helping and growing up the physical and mental health education of young people in the new era and are also the literary value of promoting the quality education of the next generation of young people in the world.

## 1. Introduction

With the continuous development of China's digital economy, China's international competitiveness has been gradually enhanced, and its international status has been steadily promoted. The development direction in the field of Chinese literature has also been gradually spread internationally. The influence of international literature communication has gradually increased. In the context of cultural communication into the world, Chinese and Western literature blend with each other. Through the integration of western excellent literature, Chinese literature also develops with the internationalization of the Internet and brings more influence. Xiaoming has many problems in the process of international communication of Chinese animation adapted from classic literature, which cannot ensure the effect of communication. We should establish a correct concept and consciousness, scientifically carry out the international communication of Chinese animation under the adaptation of classical literature, break the traditional communication mode, and lay a foundation for subsequent development [1]. New media and corresponding communication methods have played an important role by taking advantage of the special situation that epidemic lovers cannot move and gather. We have been inspired by WeChat and TikTok to improve communication concepts and methods and communication skills, enhance their effects, and accelerate the progress of Chinese culture with the assistance of the Internet and mobile Internet [2]. Haitian pointed out that the internationalization of contemporary Chinese literature is the characteristic of the new era of the great rejuvenation of the Chinese nation. Literature and art not only show quality but also conducive to the development of personal physical and mental health. Modern people should not only enrich their talents through literature and art but also cultivate life through art [3]. According to Yan and Hua, the international communication of China's core values is required by the current development. Under the implementation of the strategy, it should be carried out in full combination with the current culture. Literary works have extremely high literary value and practical significance. Taking literary works as the main body of China's core value communication effectively promotes the promotion of international status [4]. Leshi pointed out that the development of China humanities academic international exchange journals is conducive to our smooth academic exchanges with foreign countries, obtaining a large number of exchange opportunities with overseas academic scholars, and is helpful to the improvement of young people's knowledge [5]. Xingjie pointed out that there are a large number of online articles on the Internet that seriously affect the healthy growth of young people's body and mind, dispel the traditional humanistic spirit and thinking mode, and guide young people to pay more attention to Chinese literary works, carry out belief education, and enhance self-discipline consciousness, which is conducive to shaping a correct outlook on life, values, and world outlook [6]. Jie pointed out that literary education helps improve language application ability and humanistic quality. There are a large number of classic literary works in literary education. Teenagers read literary works, expand their knowledge, realize the healthy development of personal thought and spirit, improve aesthetic ability, and promote the healthy development of body and mind [7]. Xiaozhen et al. pointed out that everything has two sides, and there is no absolute good or absolute bad. When conducting mental health education for teenagers, we should first correct the values of educators and then correctly guide their mental health [8]. This study analyzes the impact of the international dissemination of Chinese literature on the physical and mental health of teenagers in the digital humanistic environment. Chinese literature is broad and profound, and each school has its own ideas. The growth of teenagers needs us to guide and dredge. Teenagers are not only the hope of the future but also the backbone of the country. The health of the people is not only the health of the body but also the health of the soul. Strengthening the health impact of literature and art is our ultimate goal. The spread of Chinese literature in the international scope is also a good education and training for domestic and foreign talents studying abroad. It spreads the advantages of Chinese literature to all parts of the world and has a long history. It affirms the value of Chinese literature and also creates positive physical and mental health for the growth of young people.

The article "Research on the Influence of International Communication of Chinese Literature on Teenagers' Physical and Mental Health in the Digital Humanistic Environment" was retracted in 2023. Reasons: signs of a paper mill; suspected computer-generated content; unreliable results or conclusions; concerns about the data.

## 2. Digital Humanities Development

In the process of the development of the Internet, it enables people to realize the interactive mode across time and space in the network world and provides a new exploration direction for Digital Humanities Research. Digital Humanities refer to the use of digital information technology to study the relevant theories and practices of humanities. Digital Humanities Research belongs to the collaborative research among interdisciplinary disciplines. Therefore, Digital Humanities Research scholars generally have multidisciplinary backgrounds, and their research results can also serve multiple disciplines. The development of Digital Humanities is so strong, mostly because of the promotion of information technology and the development of disciplines and systems in many aspects. At present, the core and boundary of Digital Humanities cannot be specifically defined. Every scholar has different views on the concept of Digital Humanities. Digital Humanities is a new subject field formed by the innovative research of traditional humanities based on modern information technology. The popularization of science and the continuous progress of information have created the current achievements of Digital Humanities. Digital Humanities has experienced more than 70 years of development. As early as the 1940s, humanistic computing was understood by people. Again, before that, someone applied computer technology to the vocabulary index to further expand the application field of computer technology. Later, more and more people began to pay attention to the relationship between computing and the humanities. In 2001, Digital Humanities was officially proposed and then received more scholars' research and attention.

## 3. Value and Significance of Chinese Literature

Chinese literature is mainly divided into classical literature, modern literature, and contemporary literature. Classical literature is mainly represented by Tang and “Song Poems” and “Four Famous Works,” modern literature is represented by Lu Xun's novels, and contemporary literature is marked by Chinese free literature with independent thoughts. Chang pointed out that with the continuous development of society and times, Chinese literary works have gone to the world, but compared with the spread of foreign literature, the internationalization process of Chinese literature is relatively slow, and Chinese culture has been upgraded to national strategy. In order to make people around the world better and faster understand Chinese literature, it is very important to find the corresponding model [9]. In Chinese classical literary novels, the author depicts their psychology and displays literary images with details and comic style strokes. This form not only enriches the character gallery of ancient Chinese literature but also shows different aspects of social life [10]. While classical literary works express human expectations, literature also lights up the spiritual lighthouse and provides humanistic care for human beings, truly reflects the purpose of “being human,” and transforms human spiritual writing into emotional power that reaches the hearts of the people. Excellent literary masterpieces are of far-reaching significance to the education of teenagers and can also drive the development of national political culture. Many excellent writers and creators are constantly writing more excellent works. It is expected that Chinese writers will inject ultimate care and profound human consciousness into their literary writing and constantly write new Chinese epics showing the progress of human spirit, marking a new height for the world literary pattern.

The article "Research on the Influence of International Communication of Chinese Literature on Teenagers' Physical and Mental Health in the Digital Humanistic Environment" was retracted in 2023. Reasons: signs of a paper mill; suspected computer-generated content; unreliable results or conclusions; concerns about the data.

## 4. The Influence of International Communication of Chinese Literature on Teenagers' Physical and Mental Health

Teenagers are the future of the motherland and the most critical period in life. This group is in a period of rapid physical and mental development. It is immature in all aspects and has a strong curiosity and thirst for knowledge, but its ability to distinguish right from wrong is weak, and its behavior is impulsive, so it is easy to blindly follow. Therefore, using literary works to convey knowledge, information, thoughts, feelings and beliefs, as well as the positive energy of all social communication activities, can effectively shape excellent ideological quality for young people. Haisong and Cheng's classical literary novel “Journey to the West” can be called a treasure of legal culture. In “Journey to the West,” mythical characters often quote laws and regulations, “FaDu,” “tiantiao,” “Tianli,” and “wangfa Tiao,” and other words with legal principles can be seen everywhere. There are more typical legal principles in the book, such as law and authority, law and rights, law and freedom, law and human feelings, law and rational desires, and law and religion [11]. Guo pointed out that classical literature education can not only enrich the connotation of Ideological and political education for college students but also improve the current situation of ideological and political education and cultivate good quality and moral quality of college students. In the process of ideological education for college students, we should pay more attention to classical literature education, enrich the experience of classical literature education, give play to the advantages of classical literature education in the process of ideological education, and establish a good foundation for teenagers' thoughts [12]. According to Xue, for international exchange students who come to China, through reading and studying Chinese literature, they can better understand China's long-standing moral and cultural level, shape their psychological healthy growth, and provide a path for the dissemination of Chinese literature [13]. In this regard, the society should pay attention to the influence of culture on the youth groups in China and create a good social environment for realizing the Chinese dream.

## 5. The Comprehensive Impact of International Communication of Chinese Literature on Teenagers' Physical and Mental Health

### 5.1. Analysis of the Characteristics of Teenagers' Physical and Mental Health in the Digital Humanistic Environment

As the young generation of the country, the education and growth of teenagers from childhood are very important, and the country attaches great importance to the cultivation of talents and school education. As a large country with a history of 5000 years of literature, China has inherited and developed its traditional culture, and many great literary works have emerged, for example, “Three Character Classic,” “Thousand Character Essay,” “Di Zi Gui,” “Tang and Song Poems,” “Four Famous Works.” In the development of digital society, the spread of Chinese literature through the Internet has far-reaching impact on the field of international literature. It also has a partial impact on the physical and mental health of teenagers. The following figure is an analysis of the characteristics of contemporary teenagers' physical and mental health:

As shown in Figure 1, in the development of digital cultural environment, teenagers' attention to physical and mental health is reflected in the shaping of personal values, social values, and world values. ldeological and political construction and cultural and educational development also have a profound impact on the growth of teenagers. The healthy growth from body to mind is the experience of the healthy growth of contemporary teenagers, which is closely related to the cultivation of talents and the future construction and development of the country. The influence of internationalization makes contemporary teenagers come into contact with more foreign cultures and arts. Under the scour of the times, the greater the influence of the development and dissemination of Chinese literature, the more important it is for shaping the physical and mental health of Chinese teenagers, and the more attention it attaches to the characteristics and inheritance of the motherland's culture.

The article "Research on the Influence of International Communication of Chinese Literature on Teenagers' Physical and Mental Health in the Digital Humanistic Environment" was retracted in 2023. Reasons: signs of a paper mill; suspected computer-generated content; unreliable results or conclusions; concerns about the data.

### 5.2. Comprehensive Analysis of Shaping Physical and Mental Health of Adolescents in Different Ages

With the progress of the Internet and the scientific level, driven by the development of the world economy, the spread of literature has also developed with the international development. Chinese literature is composed of classical literature, modern literature, and contemporary literature. China has a long history. Influenced by the region and custom culture, each place has its own unique literary achievements, which has a far-reaching impact on the international spread of China's unique literary values. The following table analyzes the impact of the international communication of Chinese literature in different ages on the physical and mental health of teenagers:

As shown in Table 1, analyzing the shaping of physical and mental health from three aspects, ideological education, physical health, and moral character shaping, we can see that with the development and progress of the times, the influence of physical and mental health of teenagers is becoming more and more important, and the achievements are also more ideal. The standard data is visualized to obtain Figure 2:

As shown in Figure 2, under the Digital Humanities, Internet technology reduces the concepts of space and time, and the cultural transmission of various countries has spread to the world with the development of Internet technology. While Chinese literature is developing towards internationalization, foreign culture is also accepted at the same time. In the education of teenagers, Chinese literature, which is fused by the combination of Chinese and Western culture, is carried forward, so that teenagers can grow at the same time. We can better understand the cultural heritage of our country and create a positive ideological construction.

### 5.3. The Influence of Chinese Literature Communication in Different Environments on Teenagers' Physical and Mental Health

The physical and mental health of teenagers can be divided into four parts from body to mind: physical health, mental health, social adaptability, and moral health. Evaluate and cultivate the growth of teenagers from different aspects. Chinese literature pays more attention to the traditional concepts of morality, intelligence, physique, beauty, and labor, such as people's ideological and political construction and the concept of respecting teachers and morality. As a country of etiquette, China has expanded its influence with the internationalization of literature, bringing better moral cultivation to more young people. The following table is obtained by analyzing the impact of the internationalization of Chinese literature dissemination on physical and mental health in different environments:

As shown in Table 2, it can be seen from the standard data that the evaluation values in the four fields of physical and mental health are higher in the digital humanistic environment. It shows that the effect of Chinese literature on youth education and cultivation is still good. The following figure is obtained by visualizing the data:

As shown in Figure 3, it can be clearly seen from the bar chart that the development of Chinese literature plays a greater role in the construction of teenagers' physical and mental health. Compared with the traditional literary environment, in the modern society of the technological globalization of the Internet, the spread of literature, accompanied by the online communication mode of the Internet, is wider and deeper. The historical allusions and fables of Chinese literature are of profound significance, which is of far-reaching significance to the quality education of teenagers and is conducive to improving moral quality and social adaptability.

The article "Research on the Influence of International Communication of Chinese Literature on Teenagers' Physical and Mental Health in the Digital Humanistic Environment" was retracted in 2023. Reasons: signs of a paper mill; suspected computer-generated content; unreliable results or conclusions; concerns about the data.

### 5.4. Compare the Coupling Degree of Adolescents' Physical and Mental Health under Different Environments

Developing Chinese literature to the world will have a far-reaching impact on the development and progress of literature for domestic teenagers. The recognition of one's own nation's literary heritage is also conducive to the cohesion of centripetal force and honor. Chinese literature has a profound foundation in terms of education and cultivation of moral quality. Through literary masterpieces of different periods, young people are also taught to learn and grow up. The following is a comparison of the coupling degree of the impact of internationalization of Chinese literature on teenagers in different environments:

As shown in Table 3, it can be seen that the coupling degree under the digital humanistic environment is higher than that under the traditional environment in terms of the impact of the development of literary communication on teenagers, and the statistical data is *T* < 10 and *P* < 0.05. The data were statistically significant. Visualize the data in the table to get the following figure:

As shown in Figure 4, modern society is a digital society, and the development of literature is also spread and influenced by new paths through the environment of digital development. For the development of Chinese literature, it can also better absorb the characteristics of foreign western literature, enhance the influence of Chinese literature, and open up a new direction for the future development of literature. To cultivate the physical and mental health of teenagers, establish correct social psychology and personal values. It also provides more capital for the training of the new generation of talents in the future.

## 6. Summary

The development of the new era is accompanied by a series of changes, which can be found from the development of literature. Chinese literature, from classical literature to modern literature and then to contemporary literature, embodies the painstaking works of literary giants in each historical period. Many Chinese literary works have more excellent definitions in terms of moral etiquette, which has more positive significance in establishing the correct values and physical and mental health of teenagers. On the one hand, it also shows the intrinsic value of Chinese literature and its value and dissemination in the field of International literature. On the other hand, as literature plays an important role in the healthy growth of young people's body and mind, it can also provide positive research value and innovative materials for the development of Chinese literature. Along with the development of literature, it also plays an important role in China's economic, artistic, educational, and social development. Chinese literature is broad and profound, and each school of thought has its own merits. Chinese literature also reflects different ideological realms. It needs positive energy guidance for the growth of young people and is an important way to cultivate future pillars of our country.

The article "Research on the Influence of International Communication of Chinese Literature on Teenagers' Physical and Mental Health in the Digital Humanistic Environment" was retracted in 2023. Reasons: signs of a paper mill; suspected computer-generated content; unreliable results or conclusions; concerns about the data.

## Figures and Tables

**Figure 1:** Analysis of the characteristics of teenagers' physical and mental health in the digital humanistic environment.

**Figure 2:** Effect analysis of internationalization of Chinese literature in different ages on shaping physical and mental health of teenagers.

**Figure 3:** An analysis of the influence of literary communication on teenagers' physical and mental health in different environments.

**Figure 4:** Analysis of the coupling degree of the influence of Chinese literature internationalization on the physical and mental health of teenagers.

**Table 1:** Effect analysis of internationalization of Chinese literature in different ages on shaping physical and mental health of teenagers (%).

Group	2000	2005	2010	2015	2020
Ideological education	35.23	41.22	51.23	57.12	71.23
Good health	41.11	53.23	64.25	67.58	73.26
Moral shaping	46.38	53.87	68.22	71.26	79.55

**Table 2:** An analysis of the influence of literary communication on teenagers' physical and mental health in different environments.

Group	Good health	Ideologically healthy	Social adaptability	Moral health
Traditional environment	42.26	46.22	50.26	53.26
Digital humanistic environment	68.38	72.2	75.26	78.28

**Table 3:** Analysis on the coupling degree of Chinese literature internationalization to teenagers' physical and mental health.

Group	The influence of internationalization of Chinese literature on teenagers' physical and mental health	
	Before coupling	After coupling
Traditional environment	45.26	51.21
Digital humanistic environment	56.13	77.76
t	7.365	8.265
P	0.035	0.020

## Data Availability

The data underlying the results presented in the study are available within the manuscript.

## References

[1] Xiaoming S. (2020). Research on the international communication of Chinese animation from the perspective of classic literature adaptation. *Media Forum*.

[2] Shenglai C. (2021). International communication of Chinese culture in the post epidemic era. *Modern communication (Journal of Communication University of China)*.

[3] Haitian Y. (2020). Historization, internationalization and nationalization of Chinese contemporary literary criticism. *Chinese Contemporary Literary Research*.

The article "Research on the Influence of International Communication of Chinese Literature on Teenagers' Physical and Mental Health in the Digital Humanistic Environment" was retracted in 2023. Reasons: signs of a paper mill; suspected computer-generated content; unreliable results or conclusions; concerns about the data.

[4] Yan Z., Hua Z. (2019). Research on the industrialization of Mo Yan's literary works and the international communication of contemporary Chinese core values. *Communication Research*.

[5] Leshi Z. (2017). The internationalization of humanities academic journals -- taking the magazine of Chinese comparative literature as an example. *Guangdong Haifeng*.

[6] Xingjie Z. (2019). The way to improve college students' online literature reading taste from the perspective of cultural confidence. *Regional Governance*.

[7] Jie C. A. I. (2021). Chinese language and literature education and humanistic quality training under the Internet. *China New Communications*.

[8] Xiaozhen G., Pingping Z., Wang M. (2021). Influencing factors and countermeasures of college students' physical and mental health education. *Shanxi Youth*.

[9] Chang L. (2022). The dilemma and way out of the translation and introduction of Chinese modern and contemporary literary works. *Science and Education Anthology*.

[10] Ximei Z. (2022). The image of miser in Chinese classical literature. *Popular Literature and Art*.

[11] Haisong J., Cheng Z. (2022). An analysis of legal propositions in Chinese classical literature -- based on the analysis of Journey to the West. *Journal of Xiangtan University (PHILOSOPHY AND SOCIAL SCIENCES)*.

[12] Guo W. (2022). Research on the influence of classical literature education on college students' ideological education. *Journal of Yanbian Institute of Education*.

[13] Xue J. (2022). Study on the reading habits of foreign students in China and the cognitive needs of Chinese literature. *Journal of Hebei North University (SOCIAL SCIENCE EDITION)*.

